# Comprehensive environmental and techno-economic feasibility assessment of biomass- solar on grid hybrid power generation system for Burdur Mehmet Akif Ersoy University Istiklal Campus

**DOI:** 10.1016/j.heliyon.2023.e22264

**Published:** 2023-11-14

**Authors:** Ercan Aykut, Bahtiyar Dursun, Sertaç Görgülü

**Affiliations:** a Istanbul Gelisim University, Faculty of Engineering and Architecture, Department of Electrical –Electronics Engineering, Avcılar, Istanbul, Turkey; b Burdur Mehmet Akif Ersoy University, Faculty of Engineering and Architecture, Department of Electrical –Electronics Engineering, Merkez, Burdur, Turkey

**Keywords:** Hybrid renewable energy systems, Techno-economic feasibility, HOMER, Renewable energy resources, Solar energy, Biomass

## Abstract

The worldwide use of clean and environmentally friendly renewable energy sources, has been increasing to prevent global warming and climate change. In this study, a hybrid renewable energy system (HRES) including biomass and solar as the source, has been investigated for Mehmet Akif Ersoy University Istiklal Campus in Burdur, Türkiye. The campus has an animal farm consisting of 300 cattle and 200 sheep. Therefore, manure of the animals will be used as the resource for biomass generation. HOMER software is used to simulate the system and to find the size and the quantity of the equipment according to the meteorological and biomass capacity of the campus. The optimum system is determined by means of net present cost (NPC) and the cost of energy (COE). In the simulation, wind energy is also investigated but since the wind speed is not sufficient to produce energy in the region, it is not considered in the optimum system. The optimum system is determined to be grid connected biomass-solar system with 5000 kW PV panels and a 1500 kW biomass generator assisted by the grid of 3000 kW. Also, the NPC of the system is estimated to be USD 18.800.000 and the COE for the system is calculated as 0,107 USD/kWh. The system also reduces the emissions causing the global warming.

## Highlights

• Renewable energy sources such as solar and biomass are utilized in this study.
• Since the university has a farm, cattle manure is used as a biomass source.
• The optimum system constitutes of biomass-solar on grid system with 1500 kW biomass generator, 5000 kW PV and 3000 kW grid.
• COE is estimated to be 0,107 USD/kWh and renewable fraction is 49,4 %.
• By using the proposed renewable system 4.554.834 kg of CO_2_, 19.746 kg of SO_2_ and 9.657 kg of NO_x_ per year is reduced.

## Nomenclature

*C*_*a,t*_: Annualized cost in total ($/year)
COE: Cost of energy
COHE: Council of Higher Education
CRF: Capital recovery factor
C_tot_: The yearly cost for the system ($/year)
E: The total expenses within the life of the project
*E*_*p,AC*_: Basic AC load power (kWh/year)
*E*_*p,DC*_: Basic DC load power (kWh/year)
*E*_*g,s*_: The amount of sales to the grid in total (kWh/year)
*f*: The rate of inflation annually
*f*_*PV*_: The derating factor for losses
*F*_0_: The fuel curve intercept
*F*_1,*io*_: The slope of the fuel curve
GHG: Greenhouse Gas
*G*_*T*_: The solar irradiance (*W*∕*m*^2^)
*G*_*Tstd*_: The irradiance at normal conditions (*W*∕*m*^2^)
HRES: Hybrid Renewable Energy System
HOMER: Hybrid Optimization Model for Electric Renewable
*I*: The total investment ($)
*i*: The percentage of real interest (%)
*i*_*0*_: The amount of nominal interest (%)
NASA: National Aeronautics and Space Administration
NPC: Net Present Cost ($)
*P*_*bio*_: The maximal generator output at minimal fossil fractions
*P*_*conv*_: The power output of the inverter (kW)
*P*_*PV*_: PV panel output power (kW)
PV: Photovoltaic
R: The total return finance
*R*_*p*_: Project lifetime (year)
ROI: The return of invest
*T*_*a*_: The outer temperature (^◦^C)
*T*_*C*_: The temperature of solar panel (^◦^C)
*T*_c_: The temperature of the solar panels at normal conditions (^◦^C)
Tp: The lifetime of the project
*x*_*fos*_: The minimal fraction of fossil fuel fraction
$U_{L}\left[\frac{W}{m^{2}K}\right]$: The Coefficient of heat transfer within the outer environment
*Y*_*bio*_: The nominal capacity of biomass generator
*Y*_*PV*_: The power of PV modules (kW)
*Z*_*bio*_: The replacement ratio of biogas against fuel
***α***: The absorbance of panels
***α***_*p*_: The temperature coefficient of power
***τ***: The transmittance coefficient of glass cover on solar panels
***ρ***_*fos*_: The density of fossil fuel
*η*_*c*_: The efficiency of electrical conversion
*η*_*conv*_: The efficiency of the inverter

## 1 Introduction

Energy is one of the most significant indicators showing the economic, environmental, and industrial development of the countries. With the increase of population, civilization and industrialization, energy demand has also been going up for decades which results in the increase of welfare. Conventional energy sources such as natural gas, oil, coal., etc. has been used worldwide for many years, however, there has been a big trend for using renewable energy sources i.e. wind, solar, hydro and biomass recently. The reason of why the use of renewable energy sources increases is their clean, sustainable, and environmentally friendly nature. Conventional sources cause emission of greenhouse gas, global warming, and climate change while the fossil fuels extract CO2 and some other gases into the atmosphere. Therefore, the use of these sources is decreasing in all around the world [[1], [2], [3], [4], [5], [6], [7]].

According to the Paris agreement made in the United Nations Climate Change Conference 2015, many countries decided to limit the carbon emissions causing the global warming and climate change. The target of the GHG emission reduction is determined to be 40 % by 2030 and 80 % by 2050. To reach this target, renewable energy sources must be replaced with the conventional ones. It is planned that 30 % of the energy will be supplied by renewables sources and in 2050, the energy is assumed to be met by completely from renewable energy sources. Therefore, the significance and the use of renewable energy is increasing worldwide. Especially power generation companies, policy makers about energy, and governments pay extra attention for this issue [8,8,9,9,10,10].

Among the significant renewable energy sources, solar energy is widely used in energy production worldwide. Being limitless, clean, and environmentally friendly makes it more charming. Besides, as well as producing energy, it is also used to provide the thermal comfort in the buildings [11].

Although being free, clean and environmentally friendly, renewable energy sources are also unstable and variable. Therefore, these sources may not be used alone. Instead, in order to achieve more efficient energy, 2 or more different energy sources i.e. solar/biomass, biomass/wind, solar/wind/hydrogen can be utilized together which is called as hybrid or combined energy system [1,2,12,13].

Studies on hybrid and combined renewable energy systems are widely encountered in the literature review.

Even though there are many different HRES studies in the literature, since the wind speed and other sources such as geothermal and hydro, are not sufficient in the region of the study, optimum system does not include theses sources. Therefore, only biomass and solar hybrid energy systems are investigated in literature review. Kumar and Channi investigated the suitability of a PV-biomass hybrid renewable energy system for a small village in India by means of economic and technical issues. The system consists of a 10 kW biomass generator, 1,1 kW PV panels 5 batteries and a 4 kW inverter. Return of invest of PV panels is about 1,5 years and the construction cost of the system within the 25 years period is estimated to be USD 21.087 [14]. Similarly, Lata- Garcia et al., evaluated solar PV/biomass hybrid system in terms of techno-economic for a house in an isolated place in the province of Guayas in Ecuador. According to the study, the load of 143 kW/day must be supplied by a 50 kW solar panels, a 28 kW biomass generator and 55 units of 140Ah batteries and a 12.5 kW inverter. The system costs USD 179.346 and the COE is estimated to be 0,253USD/kWh [15]. Another study about wind-solar-biomass hybrid energy system for the electrification of a rural area was conducted by Murugaperumal et al. They tried to determine the optimization of the energy supply of village of Korkadu, India from technical design and techno-economic aspect, in their study. The proposed HRES must meet the load of about 179 kW per day and maximum load of about 20 kW per day and the total system and power generation costs are INR 1,21 million and INR 13,71 respectively, while the performance of the battery is 36.648 kWh/year [16]. Rajbongshi et al., studied the optimization of energy supplied by grid connected solar-biomass gasifier-diesel HRES for a non-electrified district in India, for different load types and grid conditions. In the study they estimated the total COE as USD 0,145/kWh for a daily load demand of 19 kW and a maximum energy of 19 kW/day in the off-grid system condition, and if the system is grid connected, then the COE reaches about USD 0,91/kWh [17]. Similarly, Shahzad et al., proposed a gridless PV/Biomass HRES in terms of techno-economic aspect for a rural area of Punjab province in Pakistan. The optimum system consists of 10 kW solar panels, 8 kW biogas generator, 32 storage batteries and 12 kW inverter. While the initial cost is estimated to be PKR 2,64 M, total net present cost (NPC) is calculated to be PKR4,48 M. The cost of energy of the system is determined to be 5,51 PKR/kWh [18]. Also, Smruti et al., studied the optimization of a PV-biomass HRES for a house in a remote area. The system has a daily 3,6 kW peak load which is met by a PV-biomass HRES. The system has a capital cost of around 900.000 RS and the return of invest is estimated to be 12 years. If the government support of 50 % is added, then this time reduces to 6 years [19]. Kumar presented a grid connected PV-biomass HRES model for South Australia. In the study, the proposed hybrid power system is analyzed by means of an economic and environmental view. In the HRES, 200 kW PV panels, 30 kW biomass generator, 150 batteries and 200 kW inverter are used. The NPC and the COE of the optimum HRES is USD 971.377 $ and 0,129 USD/kWh respectively, and the renewable fraction is 79 % [20].

Eteiba et al., performed a study about techno economic feasibility of a PV-Biomass HRES in a rural area, in Egypt by comparing some optimization techniques such as the flower pollination, the harmony search, the artificial bee colony and the firefly algorithms. The best optimization technique for the system is found to be the firefly algorithm consisting of 24 solar panels, 4 biomass generators, and 298 batteries [21]. Bhattacharjee and Dey performed grid-connected solar/biomass hybrid system for some mills in a state, whose location is in the north-eastern region of India. According to the study, the optimum system consists of 25 kW solar panels, 6 kW biomass generator and 20 kW inverter. While the quantity of biomass material used in the system is 11.000 kg, COE and NPC is estimated to be 0,143 USD/kWh and USD78.980 [22]. Also, Kumar studied feasibility of solar/biomass hybrid power system for Auckland city, New Zealand by means of economical and clean hybrid renewable system. The modelled system includes 600 kW solar panels, 60 kW biomass generator, 800 batteries, and 600 kW inverters. 190 tons of biomass is used and the biomass generator operated 8752 h per year. The NPC and the COE of the system is calculated to be USD 1.452.058 and 0,186 USD/kWh respectively [23]. Rajanna and Saini proposed solar, biomass and biogas based integrated renewable energy systems for Karnataka, India. They analyzed the proposed renewable energy systems applying with three different scenarios based by means of NPC, COE and air polluting gas emission [24]. Ghenai and Janajreh studied solar-biomass HRES for the electrical production of Sharjah city by using micropower optimization model. They performed optimizing with sensitivity analysis of the hybrid renewable system. The annual energy production of the HRES is calculated to be 51.143.528 kWh, 74 % of which is supplied by solar system and the remaining 26 % is met by biomass system. The NPC and the COE of the HRES are calculated as USD154.901.904 and 0,328 USD/kWh respectively [25]. Gebrehiwot et al., evaluated the potential of a hybrid system for the electrification of a rural area located in Ethiopia. They determined optimum hybrid system combination with the least cost for the rural area in Ethiopia using HOMER software. The optimum system for the rural area consists of a 20 kW PV array, a wind turbine with 9 kW power, a diesel generator with 5 kW power, and 24 batteries. The NPC and COE of the system is USD 82.734 and 0,207 USD/kWh respectively [26]. Zahid et al., carried out a grid connected solar/biomass HRES model for an industrial area. Moreover, they analyzed the proposed HRES by means of techno-economic aspect. Lastly, they analyzed the grid connected biomass/solar hybrid system for different power values of the components to assess the optimum configuration with the least COE, NPC and initial cost. The proposed system constitutes of 70 MW solar panels, 7 MW biomass generator and 82,6 MW inverter. The system has a NPC of PKR 135 Billion and the COE is PKR 14,11/kW [27].

A feasibility analysis by means of technical, environmental and economic aspects has been demonstrated in this paper. The study aims to determine the optimum HRES among the biomass, solar and wind sources for Mehmet Akif Ersoy University Main campus in Burdur, Türkiye, by using HOMER. Solar radiation data was obtained from HOMER and then entered in the required section in the software. Now that the campus has a farm, cattle manure and sheep manure collected from the farm was used as biomass resource. Lastly, every combinations are evaluated according to NPC and COE and the optimum system was decided.

## 2 Methodology

As an analysis tool, HOMER computer software designed by the NREL is used to find the optimum HRES for the Istiklal Campus. HOMER is a well-known software used for the optimization, planning and the design of the hybrid systems. On grid and off grid systems can both be modelled and investigated by using HOMER. Optimization and simulation can be applied at the same time. By means of HOMER, the energy balance calculations can easily be done according to different quantity and size of the energy sources. As an input, consumed energy, wind data and solar is entered in the software and HOMER performs the sensitivity analysis. As an output, HOMER calculates NPC, COE and fuel costs. By means of HOMER software simulation, optimization and sensitivity analysis can be done easily. The block graph of HOMER is presented in Fig. 1.

**Fig. 1:** The block diagram of HOMER software.

The mathematical models of the HRES according to the sensitivity analysis and the equations of the models are as follows.

### 2.1 Model of the solar panels

The PV panel output power (*P*_*PV*_, *kW*) can be evaluated by the equation (1).

(1) $$P_{PV}=Y_{PV}f_{PV}\left(\frac{G_{T}}{G_{T_{Std}}}\right)\left[1+\alpha_{p}\left(T_{c}-T_{c,std}\right)\right]\;\left(\text{kW}\right)$$

Here, *Y*_*PV*_ (kW) stands for the power of PV modules, *f*_*PV*_ corresponds to the derating factor for losses, *G*_*T*_ (*W*∕*m*^2^) accounts for the solar irradiance, *G*_*Tstd*_ (*W*∕*m*^2^) shows the irradiance at normal conditions (1000W∕m^2^), *T*_*C*_ (^◦^C) stands for the temperature of solar panel, *T*_c,_ (^◦^C) accounts for the temperature of the solar panels at normal conditions and ***α***_*p*_ corresponds to the temperature coefficient of power [27,28].

Considering the energy balance on the solar panels, the temperature of the cell *T*_c_ can be calculated by equation (2).

(2) $$T_{c}=T_{a}+G_{T}\left(\frac{\tau \alpha }{U_{L}}\right)\left[1-\frac{\eta_{c}}{\tau \alpha }\right]\left(◦C\right)$$

Here, *T*_*a*_ (^◦^C) corresponds to the outer temperature, ***α*** stands for the absorbance of panels, ***τ*** accounts for the coefficient of transmittance for glass covering on solar panels, $U_{L}\left[\frac{W}{m^{2}K}\right]$ corresponds to the coefficient of heat transfer within the outer environment, and ***η***_*c*_ accounts for the efficiency of electrical conversion [27,28].

### 2.2 Model of the biomass generator

The biomass generator can be used in two modes. One of which is biogas and the other is fossil as a resource. Equation (3) shows the fuel consumption rate of the biomass generator.

(3) $${\dot{m}}_{bio}=Z_{bio}\rho_{fos}\left(F_{0,bio}Y_{bio}+F_{1,bio}P_{bio})(1-x_{fos}\right)$$

Here, *Z*_*bio*_ corresponds to the substitution ratio of biogas in fuel, ***ρ***_*fos*_ stands for the density of fossil fuel, *Y*_*bio*_ accounts for the nominal capacity of biomass generator, *F*_0_, corresponds to the fuel curve intercept, *P*_*bio*_ is the maximal output power of the generator for minimal fossil fuel ratio, *F*_1,*bio*_ stands for the slope of the fuel curve and *x*_*fos*_ accounts for the minimal fraction of fossil fuel fraction [27].

### 2.3 Model of the inverter

To convert DC voltage produced by solar panels to supply AC loads, a one directional inverter is used. Equation (4) shows the overall capacity of the inverter according to the efficiency.

(4) $$P_{conv}=P_{PV}\eta_{conv}\left(\text{kW}\right)$$

Here, *P*_*conv*_ corresponds to the power output of the inverter, *P*_*PV*_ stands for the DC power input to inverter and ***η***_*conv*_ accounts for the efficiency of the inverter which is assumed to be 0,85.

### 2.4 Model of the costs

In order to determine the feasibility of the HRES, NPC, COE and the return of invest of the system must be calculated.

#### 2.4.1 Net present cost

NPC is achieved by subtracting total incomes from the total costs within the life of the project.

Initial cost, replacement cost, O&M cost, fuel cost and electricity buying cost can be included in the costs where the selling of energy to the grid is classified under incomes.

The calculation of NPC is given in equation (5) [1,29]:

(5) $$NPC=\frac{C_{tot}}{CRF\left(i,T_{p}\right)}$$

Here, C_tot_ ($/year), stands for annual cost of the system *i* (%), accounts for the interest rate, Tp, and CRF correspond to the lifetime of the project, and the capital recovery factor [30].

#### 2.4.2 Cost of energy

COE is defined as the average cost of 1 kWh of electrical energy generated by the system. Equation (6) presents the calculation of COE [1,29,30].

(6) $$\frac{C_{a,t}}{E_{p,AC}+E_{p,DC}+E_{g,s}}$$

Here E_p,AC_ stands for alternative current basic load (kWh/year), E_p,DC_ accounts for direct basic load (kWh/year) and E_g,s_ accounts for total sales amount to the grid (kWh/year).

#### 2.4.3 Return of invest

The return of invest (ROI) can be evaluated by using equation (7). Here, *I* stands for the investment in total, R accounts for the total return amount and E corresponds to the expenses in total within the life of the project [27].

(7) $$ROI=\frac{I}{R-E}$$

## 3 Material and methods

### 3.1 Load assessment

The campus for which the study is made, is located in Burdur, northeastern of Mediterranean region, whose latitude is 37.7144° N and altitude is 30.2715°E. The campus is located at the 37° 42′ 51.9948″ and 30° 16′ 17.7132″ coordinates [31]. The student population of the campus is about 32.000 [32]. A view from the satellite for the campus can be seen in Fig. 2.

**Fig. 2:** A view from the satellite for the location of the University Campus.

The current electrification of the campus is provided by the grid. The consumed energy data of the campus are obtained from CK Akdeniz Electric [33]. According to the load demand data, it can be seen that the peak load is 2189,53 kW and the load varies between 798,21 kWh and 2189,53 kWh, while the daily total load demand is about 34 MWh. The load demand of the campus within a day is shown in Fig. 3.

**Fig. 3:** Daily load demand of the Istiklal campus.

The load demand has its minimum amount between the hours 06:00 and 07:00 because the outer lighting is turned off, and the load demand has the highest rate between 17:00 and 20:00 since there are evening courses in the campus.

### 3.2 Potential of the resources

Even though there are many different HRES studies in the literature, since the wind speed and other sources such as geothermal and hydro, are not sufficient in the region of the study, optimum system does not include theses sources. Therefore, only biomass and solar Hybrid energy systems are investigated in the study.

#### 3.2.1 Potential of solar energy

The insolation data of the campus is obtained by HOMER software which gets the information from NASA. The data are compared with renewable energy directorate and found to be nearly same. The insolation data is used accordingly [34]. Fig. 4 shows the solar energy density as per months. According to the graph, the solar energy density is 5,85 kWh/m^2^ per day in a year and from the graph, also the average of the clearness index is 0,621.

**Fig. 4:** Density of solar energy and clearness index for the campus.

#### 3.2.2 Potential of biomass energy

Burdur is a significant city suitable for farming and animal feeding. Therefore, the Council of Higher Education (COHE), designing and managing the universities and the institutes, authorized Burdur Mehmet Akif Ersoy University in the regional development focused mission differentiation and expertizing program [35]. In this context, the university established a research and application center and an animal farm including 160 cattle and 100 sheep. So, the manure of the animals in the farm will be used as a biomass resource in this study. For biomass data, the animal count has been received from the farm and the manure quantity has been calculated according to the information from the literature review. According to literature review, one cattle produces 15 kg manure per day which corresponds to 2400 kg daily production for the farm and also, one sheep gives 0,5 kg manure per day which means 50 kg per day [[36], [37], [38]]. Therefore, the daily total manure production of the farm is 2,45 tons. The monthly feedstock production of the farm is presented in Fig. 5.

**Fig. 5:** The feedstock quantity of the farm produced in months.

### 3.3 Components and the used in the HRES

In the study, it is aimed to propose a HRES instead of current conventional system. As a renewable resource, biomass, solar hybrid system is proposed. In the case of the renewable sources are limited then grid will contribute to the continuity of the electrification and according to availability and sufficiency of the sources, the optimum system is determined by using HOMER [39]. The components utilized in the suggested system are presented in Fig. 6.

**Fig. 6:** The components used in the proposed system.

It is important to choose the correct size and types of the components to meet the load demand.

#### 3.3.1 Solar panel

The solar panels used in HOMER is determined to be 1 kW with 12V DC output. Since solar panels cannot produce energy at night, the HRES will be assisted by the other sources. The solar panels are simulated between 0 kW and 12500 kW. Generic flat plate PV model solar panel is used in the study [40]. The technical and economic specifications of the solar panels is presented in Table 1.

**Table 1:** The techno-economical specifications of the solar panels.

Parameter	Value	Unit
Initial cost	600	USD
Replacement cost	600	USD
O&M cost	10	USD
Life	25	years
Nominal power	1	kW

#### 3.3.2 Biomass generator

In the study, biomass generator is proposed to assist the PV panels. In HOMER Generic biogas genset biomass generator is used and simulated between 0 kW and 8000 kW [30]. The technical and economic specifications of the solar panels is presented in Table 2.

**Table 2:** The technical and economic data of the biomass generator.

Parameter	Value	Unit
Initial cost	2450	USD/kW
Replacement cost	2450	USD/kW
Operational and Maintenance cost	0,10	USD/hour
Lifetime	20000	hours
Nominal power	1500	kW

#### 3.3.3 Inverter

The simulation is made for the inverter with the power between 0 and 7500 kW. The capital cost and replacement cost ABB MGS 100 model inverter are USD 100/kW and USD 100/kW respectively where the operational cost is neglectable. Additionally, the inverter has the efficiency of 90 % [41].

#### 3.3.4 Grid

In case the produced energy from the renewable sources is not enough to supply the load, grid will be used to maintain the sustainability of the energy supply. Grid is simulated for the values 0 and 3000 kW and the capacity of sale is determined as 1000 kW.

## 4 Results and discussions

The purpose of the analysis is to decide which is the most feasible hybrid energy sources with minimum COE and NPC, among PV and biomass. In the study the energy source data and the load data were entered and by using HOMER the optimum system, parameters were determined [39].

### 4.1 Analysis of optimum system

Among the renewable energy sources, wind, geothermal and hydroelectric potential is not enough to produce energy, and solar potential is high, and the campus has an animal farm, the campus has also biomass potential. In case the solar and biomass production may not be enough, grid option is also included in the proposed system. HOMER presented a few options from which the optimum system can be determined. The system having the least COE constitutes of a grid connected Biomass system. The COE of this system is calculated as USD 0,119/kW and the NPC of the system is USD 19.600.000. Moreover, there is another option consisting of a grid connected biomass-solar system. The COE and the NPC of this system is USD 0,107/kW and USD 18.800.000 respectively. Since the COE of the latter system is lower, it can be preferred as the optimum system because it is more environmentally friendly and cleaner. The values of the components of the system such as PV, biomass, inverter, grid, COE, NPC, the operating hours of biomass generator and biomass quantity used in the system can be seen in Table 3.

**Table 3:** Parameters of the optimum configuration of the system for the campus.

PV (kW)	Bio (kW)	Grid (kW)	Inverter (kW)	Cost/NPC ($)	Cost/LCOE ($/kWh)	Cost/Operating cost ($/yr)	Bio Hours	Bio/Production (kWh)	Bio/Fuel (tons)
0	1500	3000	0	19,6 million	0.119	1.233.100	287	430.500	1292
5000	1500	3000	5000	18,8 million	0.107	728.083	152	227.735	683

According to the analysis, considering the optimum system, the average biomass quantity and average solar global irradiance are nearly 2,45 tons/day and 5,85 kWh/m^2^ per day, respectively for the campus. The optimum system constitutes of 5000 kW PV and inverter, 1500 kW biomass and 3000 kW grid.

### 4.2 Power production of the system

In the optimum system, PV panels produced 7.287.876 kWh/year while the biomass generator produced 227.735 kWh/year and grid was used for 6.924.194 kWh/year. Total produced energy of the hybrid system is 14.439.806 kWh/year. Considering these values, the renewable fraction is calculated to be 49,4 %. The system used 683 ton biomass as a fuel and biomass generator worked 152 h per year. Fig. 7 shows the average production of electrical energy.

**Fig. 7:** Monthly average electrical power produced by the proposed system for the campus.

Economic analysis is also made by HOMER and the according to the analysis the initial cost of the optimum hybrid system is USD 9.425.000, the COE energy is USD 0,107/kW and the operational cost is USD 941.123. Compared with the present grid connected system, the COE of the suggested system is nearly same as the system consisting of only grid at the beginning but considering the environmental parameters and the return of investment, the proposed system will be a better choice. Excess energy to be sold to the grid is estimated to be 582.519 kWh/year which corresponds to the 4,03 % of the produced energy.

### 4.3 Emission of the system

In the production of energy, currently, fossil fuel-based energy systems are used. These fossil fuels emit some kinds of gases polluting the air and causing the global warming. Replacing conventional energy sources with the environmentally friendly renewable energy sources reduce these emissions. In this proposed study, by using renewable energy sources, it is aimed to reduce the gas emissions. The emission values of the proposed hybrid system and the emission from the grid is compared and presented in Table 4. The only grid system emits 8.931.048 kg of CO_2_, 38.718 kg of SO_2_ and 18.936 kg of NO_x_ per year while the renewable system emits 4.376.214 kg of CO_2_, 18.972 kg of SO_2_ and 9.279 kg of NO_x_ per year. According to the Table 4, CO_2_, SO_2_ and NO_x_ amount of the system is much lower than only grid system. The reduction is 4.554.834 kg of CO_2_, 19.746 kg of SO_2_ and 9.657 kg of NO_x_ per year.

**Table 4:** Gas Emissions of grid and the hybrid renewable system.

Quantity	Only from grid	From renewable energy	Difference in Emissions
Carbon Dioxide (CO_2_)	8.931.048 kg/year	4.376.214 kg/year	4.554.834 kg/year
Sulfur Dioxide (SO_2_)	38.718 kg/year	18.972 kg/year	19.746 kg/year
Nitrogen Oxides (NO_x_)	18.936 kg/year	9.279 kg/year	9.657 kg/year

### 4.4 Sensitivity analysis

Because the data of the renewable energy sources like solar and biomass are variable, the sensitivity analysis is made to determine the economic parameters. The biomass quantity values are 2,45, 5, 10, 20 tons/day and the solar radiation value varies between 4,85 and 7,85 kWh/m^2^/d. The result of sensitivity analysis can be seen in Table 5.

**Table 5:** Result of the sensitivity analysis.

Solar Scaled Average (kW/m^2^/day)	Biomass Scaled Average (tons/day)	PV (kW)	Bio (kW)	Grid (kW)	Converter (kW)	NPC ($)	LCOE ($/kWh)	Operating Cost ($/year)	Ren. Factor (%)	Total Fuel (tons/year)	Production (kW)	O/M Cost ($/year)
4,85	2,45	2.500	1.500	3.000	2.500	19,5 M	0,118	1,01 M	23,1	773	257.735	25.800
5,85	2,45	5.000	1.500	3.000	2.500	18,8 M	0,107	728.083	49,4	683	227.735	22.800
6,85	2,45	5.000	1.500	3.000	2.500	18,6 M	1,104	711.192	50,6	683	227.735	22.800
7,85	2,45	5.000	1.500	3.000	2.500	18,5 M	0,103	704.252	51,1	683	227.735	22.800
4,85	5,00	2.500	1.500	3.000	2.500	19,5 M	0,118	1,01 M	23,1	778	259.500	25.950
5,85	5,00	5.000	1.500	3.000	2.500	18,8 M	0,107	728.142	49,4	688	229.500	22.950
6,85	5,00	5.000	1.500	3.000	2.500	18,6 M	1,104	711.250	50,6	688	229.500	22.950
7,85	5,00	5.000	1.500	3.000	2.500	18,5 M	0,103	704.310	51,1	688	229.500	22.950
4,85	10,00	2.500	1.500	3.000	2.500	19,5 M	0,118	1,01 M	23,1	778	259.500	25.950
5,85	10,00	5.000	1.500	3.000	2.500	18,8 M	0,107	728.142	49,4	688	229.500	22.950
6,85	10,00	5.000	1.500	3.000	2.500	18,6 M	1,104	711.250	50,6	688	229.500	22.950
7,85	10,00	5.000	1.500	3.000	2.500	18,5 M	0,103	704.310	51,1	688	229.500	22.950
4,85	20,00	2.500	1.500	3.000	2.500	19,5 M	0,118	1,01 M	23,1	778	259.500	25.950
5,85	20,00	5.000	1.500	3.000	2.500	18,8 M	0,107	728.142	49,4	688	229.500	22.950
6,85	20,00	5.000	1.500	3.000	2.500	18,6 M	1,104	711.250	50,6	688	229.500	22.950
7,85	20,00	5.000	1.500	3.000	2.500	18,5 M	0,103	704.310	51,1	688	229.500	22.950

According to the analysis, as of the current average values of 5,85 kWh/m^2^/d solar radiation and 2,45 ton/day biomass quantity, the optimum system consists of grid connected biomass-solar system. This configuration seems the best choice from the renewable sources. The increase in the solar radiation also affects the solar energy produced directly. Similarly, as the quantity of biomass increases, energy produced from biomass will also go up.

## Conclusions

By using renewable energy sources, the emissions of the hazardous gases causing the global warming, can be reduced. A biomass-solar on grid hybrid system is modelled according to environmental and techno economical aspects for Burdur Mehmet Akif Ersoy University Istiklal campus. Since the university has an animal farm, biomass energy from the animal manure is considered to minimize the fuel cost. According to the outputs of the analysis made by HOMER computer software,

The optimum system constitutes of biomass-solar on grid system with 1500 kW biomass generator, 5000 kW PV and inverter and 3000 kW grid. Besides, the optimum system has the NPC of USD 18.800.000 while the COE is estimated to be 0,107 USD/kWh. In addition, 2,45 tons of manure can be used daily. The initial cost of the system is evaluated to be USD 941.123.

Excess energy sold to the network is calculated to be 582.519 kWh/year which corresponds to 4,03 % of the produced energy. Renewable fraction is 49,4 %. Also, by using the proposed renewable system 4.554.834 kg of CO_2_, 19.746 kg of SO_2_ and 9.657 kg of NO_x_ per year is reduced. The project life is determined as 30 years. Since the university has a farm, cattle manure is used as biomass source to produce energy. So, in other universities having similar conditions, biomass energy production may be a good solution to produce cleaner energy.

The results of the analysis demonstrate that the suggested system has a lower COE compared with the current fossil-based grid system. Another advantage of the proposed system is that it is cleaner and less pollutant. By using the system CO_2_ and other emissions will be reduced in parallel with the Paris agreement conditions. Since the wind speed is not sufficient for the energy production in the campus, it is not considered in this study.

In the future work, other places can be examined by means of the renewable energy sources or other energy source opportunities may be considered for the university campus.

## Funding

This research did not receive any specific grant from funding agencies in the public, commercial, or not-for-profit sectors.

## Data availability

The data will be available on request.

## Additional information

No additional information is available.

## Ethics declaration

Informed consent was not required for this study because there is no study on humans or animals.

## CRediT authorship contribution statement

**Ercan Aykut:** Writing – original draft, Supervision, Formal analysis, Data curation, Conceptualization. **Bahtiyar Dursun:** Writing – original draft, Visualization, Project administration, Methodology, Data curation, Conceptualization. **Sertaç Görgülü:** Writing – review & editing, Writing – original draft, Validation, Investigation, Data curation, Conceptualization.

## Declaration of competing interest

The authors declare that they have no known competing financial interests or personal relationships that could have appeared to influence the work reported in this paper.
